# Spatial-Temporal Evolution and Influencing Factors of Urban Green Innovation Efficiency in China

**DOI:** 10.1155/2022/4047572

**Published:** 2022-06-11

**Authors:** Chengwu Lu, Min Chen, Guixian Tian

**Affiliations:** ^1^School of Business, Zhejiang Wanli University, Ningbo, China; ^2^School of Business, Wenzhou University, Wenzhou, China; ^3^School of Business, Pingxiang University, Pingxiang, China

## Abstract

Promoting green urban development has become a common consensus to address environmental pollution and ecological damage, but we know little about the measurement and drivers of urban green innovation efficiency (GIE). In this article, firstly, we established a framework for assessing urban green innovation efficiency through multidimensional data, then used the spatial econometric model to reveal the spatiotemporal evolutionary characteristics of urban GIE, and, finally, analyzed the influencing factors and spatial spillover effects of urban GIE. The results show the following: (1) The overall urban GIE in China was low and had significant spatial agglomeration, mainly concentrated in the Yangtze River Delta and Pearl River Delta regions with spatial locking characteristics, while the GIE of cities in undeveloped regions does not change much. (3) There was much room for improvement in the input-output system of green innovation, considering that the sources of inefficiency in most cities were insufficient investment in scientific and technological innovation personnel and innovation environment, excessive environmental pollution, and limited technological output. (4) Foreign direct investment, financial development, and manufacturing industry agglomeration had positive effects on urban GIE. These research findings and policy implications are of certain reference value for other emerging developing countries to implement urban governance and green development.

## 1. Introduction

Since the reform and opening up, China's urbanization has made remarkable achievements. The urbanization rate has increased from 17.9% in 1978 to 58.5% in 2017. It took China 40 years to go through the urbanization process on which the developed countries spent hundreds of years. However, the rapid urbanization has also brought great pressure to the ecological environment of the city, resulting in serious pollution problems [1, 2]. In order to solve these problems, the Chinese government has put forward the strategy of ecological civilization construction and green innovation development. Under the background of global green economic transformation, urban development has entered a new development mode driven by innovation and constrained by resources and environment [3, 4]. Therefore, improving the efficiency of green innovation is an important way to achieve the goal of global sustainable development.

So far, academia has not given a definition of green innovation that can be understood and widely accepted by the public. In general, the concept of green innovation (GI) is similar to that of the environmental innovation and ecological innovation. Green innovation usually refers to the adoption of new or improved processes, technologies, practices, systems, products, etc. by companies in order to reduce and avoid environmental damage [5, 6]. In a broad sense, green innovation also includes technological innovation, institutional innovation, and cultural innovation that promote sustainable economic, ecological, and social development [7–9]. Green innovation efficiency (GIE) refers to the performance in the development of green innovation. It is generally believed that GIE is to bring environmental benefits into the process of innovation input and output and obtain the optimal innovation output at the lowest cost of resources and environment [10, 11]. How to measure the efficiency of green innovation scientifically has been a hot issue in environmental economics. Although many studies have used different methods to measure the GIE of enterprises and industries, how to measure the efficiency of urban green innovation has been stagnant. In addition, we still know little about the driving factors of urban GIE.

The efficiency of urban green innovation is closely related to the environmental regulation, human capital, industrial structure, financial development, and other factors, which may jointly affect and even determine the process of urban green innovation development to a certain extent [12, 13]. At the same time, since the knowledge spillover effect has the distance decay effect, the GIE of a city will be affected by the neighboring cities [14, 15]. Such knowledge spillover will affect the spatial distribution characteristics and evolution pattern of urban GIE and bring about a wider range of changes in the economic pattern. Therefore, it is necessary to explore the spatial-temporal characteristics and influencing factors of urban GIE. This paper takes the city as the research unit, and from the input-output perspective, it tries to (1) obtain the spatial-temporal evolution characteristics of GIE of Chinese cities; (2) analyze the sources of urban GIE inefficiency in terms of the structure of inputs and outputs; (3) understand how the environmental regulation, industrial agglomeration, financial development, and foreign direct investment affect the efficiency of urban GIE, and what the spatial spillover effect of these factors is.

Compared with the previous literature, the main contributions of this paper are as follows: First, we constructed a set of relatively perfect evaluation indicators of urban GIE and used the Undesirable-SBM model to measure the GIE of Chinese cities. Compared with the previous studies using a single indicator, it can measure the efficiency of green innovation more comprehensively. Second, from the perspective of spatial interaction, we used the spatial econometric model to explore the driving effect of environmental regulation, industrial agglomeration, financial development, and foreign direct investment on GIE, which enriches the theoretical research on the influencing factors of urban GIE. Third, the research methods and conclusions of this paper are of great enlightenment value for the urban environmental governance and urban sustainable development in other developing countries.

The remainder of this paper is structured as follows: The related literature on green is described in Section 2. In Section 3, we introduced the indicators of urban GIE assessment and described the variables and spatial econometric models for regression analysis. In Section 4, we reported the results of this paper. Our research focused on three parts: spatial and temporal variation characteristics of urban GIE in China, inefficiency decomposition of input-output indicators of urban GIE, driving factors, and spatial spillover effects of urban GIE. In Section 5, we summarized the main findings and discussed some potential avenues for further research.

## 2. Literature Review

As the world's environmental pollution constantly increases and the energy crisis intensifies, there is a consensus to promote the environmental improvement by increasing the level of green innovation. Since the 1990s, more and more research studies have focused on how to reduce negative environmental impacts through green innovation, and scholars from different disciplines have studied green innovation from different perspectives, such as environmental economics [16], innovation economics [17], and strategy management [18]. The relevant researches can be summarized as follows.

Green innovation efficiency measurement methods: in order to obtain more accurate evaluation results, the evaluation methods of GIE are also developing. There are many methods used in the existing research: (1) *Single Indicator Method*. It takes the output of green innovation as the index to measure the efficiency of green innovation. Among them, the commonly used index is the green patent [19, 20]. (2) *Comprehensive Indicator Method*. Green innovation activities involve a wide range, so a single index obviously cannot cover most of the green innovation factors. Therefore, much existing literature selected a number of indicators, from the green innovation input to environmental performance, to form a comprehensive evaluation index to measure the efficiency of green innovation [21, 22]. (3) *Input-output Analysis Method*. The most widely used methods are stochastic frontier analysis (SFA) and data envelopment analysis (DEA). In specific empirical studies, DEA and SFA mainly measure the GIE of industries and regions. For example, Fang et al. [23] used the nonradial distance function data envelopment analysis (DDF-DEA) to evaluate the green innovation efficiency of China's high pollution industries. Liu et al. [24] utilized SBM-DEA to measure the green innovation efficiency of China's high-tech industries. Lin et al. [25] used DEA window analysis to measure the green innovation efficiency of China's manufacturing industry. Long et al. [26] measured the efficiency of green innovation in 30 provinces of China through EPSi-based measurement (EBM) and Malmquist Luenberger.

(2) Influencing factors of green innovation efficiency: compared with the traditional innovation, the spillover effect of green innovation can achieve a “win-win” result with both economic development and environmental benefits [27]. Therefore, it is very important to explore the driving forces of green innovation, especially the differences between green innovation and traditional innovation [28, 29]. The existing research studies on the influencing factors of green innovation can be summarized in three aspects: (1) *Technological Innovation Capability*. The innovation capability of enterprises is an important factor to improve the innovation efficiency. However, relevant studies have found that because green innovation technology has the nature of public goods, enterprises with technological advantages generally tend to improve the traditional innovation efficiency rather than the GIE [30–32]. (2) *Market Demand Factors*. Consumer demand for environmentally friendly products and clean technologies is an important driving force for green innovation in enterprises [33, 34]. At present, the global market demand is moving towards low-pollution, low-energy products, and processes, and companies are paying more and more attention to providing green and low-carbon products and services to consumers. The development of environmental awareness is an important driving force to promote the GIE. (3) *Institutional Factors*. Due to the negative externality of environmental problems, green innovation, as a public product, has a relatively weaker market driving force than the traditional innovation, which makes the environmental regulation one of the main factors of green innovation. “Porter Hypothesis” asserts that the environmental regulation will force enterprises to improve their green innovation ability, reduce environmental pollution, and improve their economic benefits [35]. For example, a large number of studies have pointed out that the role of environmental regulation in green innovation has the heterogeneity effect on industries, regions, and firms [36–38]. In addition, the organizational system, R&D investment, and management strategy also have an impact on the efficiency of green innovation [39, 40]. With the continuous development of spatial economics, the spatial autocorrelation of green innovation has gradually been paid attention to by empirical research [41–43], and relevant research studies have begun to use spatial econometric model to explore the impact of industrial structure, educational capacity, infrastructure, environmental policies, and other factors on GIE. For example, Luo and Zhang [44] found that the education level and maturity of technology market had significant positive correlation with regional GIE. Huang and Wang [45] showed that the improvement of transportation infrastructure could improve the efficiency of regional green innovation.

## 3. Methodology and Data

### 3.1. Methodology

#### 3.1.1. Undesirable-SBM Model

Generally, there are two basic DEA models to measure the efficiency of green efficiency. One is the radial DEA model. But it has a disadvantage that it ignores the relaxation of input-output variables, which leads to errors in the estimation results. The other is the nonradial DEA model. It overcomes the shortcomings of the traditional radial DEA model and can measure the efficiency value more accurately, but it is difficult to calculate. This paper adopted the Undesirable-SBM model proposed by Tone [46] to measure the efficiency of urban GIE in China. The calculation formula is as follows:

(1) $$\begin{array}{c} \min p=\frac{1-1/m\sum_{i=1}^{m}Si_{i}^{-}/x_{i0}}{1+1/S_{1}+S_{2}\left(\sum_{r=1}^{S_{1}}S_{r}^{g}/y_{r0}^{g}+\sum_{r=1}^{S_{2}}S_{r}^{b}/y_{r0}^{b}\right)}, \end{array}$$

(2) $$\begin{array}{c} \text{subject to}\left\{\begin{array}{c} x_{0}=X\gamma +S^{-},\\ y_{0}^{g}=Y^{g}\gamma -S^{g},\\ y_{0}^{b}=Y^{b}\gamma -S^{b},\\ S^{-}\geq 0,S^{g}\geq 0,S^{b}\geq 0, \end{array}\right) \end{array}$$

In formula (2), *p* is the efficiency value, *m*, *s*_1_, and *s*_2_ respectively, represent the number of input variables, desirable output variables, and undesirable output variables;  *x*_0_, *y*_0_^*g*^, and *y*_0_^*b*^ are the eigenvectors of input variables, desirable output variables, and undesirable output variables; *X*, *Y*^*g*^, and *Y*^*b*^ are the relationship matrix of input variables, of desirable output variables, and undesirable output variables, respectively; *S*^−^, *S*^*g*^, and *S*^*b*^ represent the relaxation of input variables, desirable output variables, and undesirable output variables in the Undesirable-SBM model; and *γ* is the weight matrix of the decision-making unit (DUM). The range of the efficiency value calculated by the undesirable-SBM model is 0 < *p* ≤ 1; only when *p*=1, it indicates that the DMU is effective, otherwise, ineffective.

The advantage of the Undesirable-SBM model is that it cannot only measure the value of GIE of each DUM but also decompose whether the insufficient desirable output variables, the redundant input variable, or the undesirable output variables are the sources of the inefficiency of DUM. Therefore, it can provide direction for improving the efficiency of each DUM based on the input-output structure. In the objective function in formula (1), the three relaxation variables *S*^−^, *S*^*g*^, and *S*^*b*^ follow the decreasing law. When *S*^−^=*S*^*g*^=*S*^*b*^=0, the efficiency value *e*=1 and the value of the model function reaches the optimal solution. When *e* < 1, it indicates that there is efficiency loss in the DUM. We decomposed the sources of inefficiency into the following functions:

(3) $$\begin{array}{c} \text{inefficiency source}=\left\{\begin{array}{c} {\text{IE}}_{\text{input}}=\frac{1}{2m}\overset{m}{\underset{i=1}{\sum }}\frac{Si_{i}^{-}}{x_{i0}},\\ {\text{IE}}_{\text{output}}\frac{1}{S_{1}}\overset{S_{1}}{\underset{r=1}{\sum }}\frac{S_{r}^{g}}{y_{r0}^{g}},\\ {\text{IE}}_{\text{bad}-\text{output}}\frac{1}{S_{2}}\overset{S_{2}}{\underset{r=1}{\sum }}\frac{S_{r}^{b}}{y_{r0}^{b}}, \end{array}\;\right. \end{array}$$

Here, IE_input_ represents the inefficiency decomposition of input variables, IE_output_ is the inefficiency decomposition of desirable output variables, and IE_bad−output_ is the inefficient decomposition of undesirable output variables. The meaning of other variables is consistent with that in equation (1).

#### 3.1.2. Spatial Autocorrelation Analysis

Tobler's first law of geography points out that the spatial autocorrelation of things is closely related to distance [47]. In order to explore the spatial characteristics of urban green innovation efficiency, this paper used Global Moran's I index and local Getis-Ord Gi*∗* index in Exploratory Spatial Data Analysis [48] to analyze the spatial autocorrelation of GIE.

This paper used Global Moran's I index to explore the overall spatial autocorrelation of attribute values in the region, so as to judge the spatial agglomeration status of urban GIE.

(4) $$\begin{array}{c} \text{Moran's I}=\frac{n\sum_{i=1}^{n}\sum_{j=1}^{n}W_{ij}\left(X_{i}-\bar{X}\right)\left(X_{j}-\bar{X}\right)}{\sum \left(X_{i}-\bar{X}\right)\sum_{j=1}^{n}W_{ij}}, \end{array}$$

Here, *n* is the sample size of the study. *X*_*i*_ and *X*_*j*_ are the GIE values of city *i* and city *j*, respectively, $\bar{X}$ is the average efficiency value of the sample, and *W*_*ij*_ is the spatial weight matrix between cities. In order to more accurately measure the distance decay characteristics of green innovation spillover, we used the reciprocal of geographical distance between cities as the spatial weight matrix.

We used the Getis-Ord Gi*∗*index to analyze the spatial heterogeneity of local regions. It can reflect the aggregation of regions of high or low values in space, so as to identify the hot and cold points with statistical significance.

(5) $$\begin{array}{c} G_{i}^{*}\left(d^{2}\right)=\frac{\sum_{j=1}^{n}W_{ij}X_{j}-\bar{X}\sum_{j=1}^{n}W_{ij}}{\sqrt{\sum_{j=1}^{n}X_{j}^{2}/n-{\bar{X}}^{2}}\sqrt{\left[n\sum_{j=1}^{n}W_{ij}^{2}-{\left(\sum_{j=1}^{n}W_{ij}\right)}^{2}\right]/n-1}}, \end{array}$$

where *X*_*j*_ is the GIE value of city *j*, *W*_*ij*_ is the spatial weight matrix, and $\bar{X}$ is the average value of GIE of all samples *j*.

#### 3.1.3. Spatial Econometric Model

In order to overcome the problem that the traditional econometric model ignores the spatial heterogeneity, this paper used the spatial econometric model to explore the influencing factors of urban GIE. Based on the research of Elhorst [49], this paper set up three spatial econometric models: Spatial Lag Model (SLM), Spatial Error Model (SEM), and Spatial Durbin Model (SDM). The corresponding model setting and spatial interaction effects of the three basic models are as follows.

*Spatial Lag Model (SLM)*. The model setting is that the dependent variables are not only affected by their own explanatory variables, but also by the interregional explanatory variables.

(6) $$\begin{array}{c} Y_{it}=\rho \sum_{j=1}^{n}W_{ij}Y_{it}+\beta_{k}x_{it}+\mu_{i}+\gamma_{it}+\varepsilon_{it}. \end{array}$$

Here, *i* represents the research unit, *i*=1,2,3,…, *N*, *t* is the research period, *W*_*ij* _ represents the spatial weight matrix, *Y*_*it*_ represents the dependent variable, *ρ* is the spatial autoregressive coefficient, *x*_*it*_ represents the independent variable, *β*_*k*_ is the coefficient of the corresponding independent variable regression, *μ*_*i*_ represents the spatial fixed effect, *γ*_*it*_ represents the time fixed effect, and *ε*_*it*_ is the error term.

*Spatial Error Model (SEM)*. In the process of model setting, there is a spatial autocorrelation in the error term, that is, the error term in one space may have spatial spillover effect on the other regions.

(7) $$\begin{array}{c} Y_{it}=\beta_{k}x_{it}+\mu_{i}+\gamma_{it}+\varphi_{it}, \end{array}$$

(8) $$\begin{array}{c} \varphi_{it}=\partial \sum_{j=1}^{n}W_{ij}\varphi_{it}+\varepsilon_{it}. \end{array}$$

Here, *φ*_*it*_ is the error term of spatial autocorrelation and *∂* is the spatial autocorrelation regression coefficient of disturbance term.

*Spatial Durbin Model (SDM).* SLM and SEM could not explain the endogenous interaction effect or the spatial interaction effect with spatial autocorrelation error term. Therefore, Pace and Lesage thought that it could be further enhanced by using SDM.

(9) $$\begin{array}{c} Y_{it}=\rho \sum_{j=1}^{n}W_{ij}Y_{it}+\beta_{k}x_{it}+\sum_{j=1}^{n}W_{ij}x_{jt}\delta +\mu_{i}+\gamma_{it}+\varepsilon_{it}. \end{array}$$

Here, *δ* is a parameter vector of *k* dimension and the meaning of the other parameters is consistent with that in formula (6).

### 3.2. Index System and Variables

#### 3.2.1. Modified Evaluation Index of Urban GIE

The biggest difference between green innovation and traditional innovation is that the former not only pursues economic benefits but also takes the environmental protection into account. Therefore, it is necessary to measure the efficiency of urban green innovation and introduce relevant variables of environmental pollution. We regarded the urban green innovation as an input-output process analysis and treated the environmental pollution as an undesirable output. Considering the availability and uniformity of data, the input-output index system we established is shown in Table 1.

1. Green innovation inputs: according to the endogenous growth theory [50], innovation inputs generally contain the innovation capital, labor, and knowledge stock. Besides, since the innovation infrastructure is crucial for innovation, we also considered the innovation environment inputs, and in this paper, they are the cultural environment and the information network environment.
2. Green innovation outputs: green innovation outputs include the direct technological outputs and economic effects brought by innovation. In the current literature, the green patent is the most widely used indicator to measure green innovation; the economic output is expressed in per capita GDP.
3. Undesirable outputs: the environmental pollution is undesired in the green innovation process; therefore, we took the environmental pollutant emission of the city as the undesirable output index of green innovation. Based on the calculation method of Bai et al. [51], we assigned the industrial waste gas emission, industrial wastewater emission, and industrial fixed waste emission of the city with weights of 0.3, 0.4, and 0.3, respectively, and obtained the comprehensive environmental pollution index of the city through weighted calculation.

#### 3.2.2. Influential Factors on Urban GIE

The efficiency of urban green innovation is the result of multiple factors. This paper analyzed the influencing factors and spatial spillover effect of urban GIE from the aspects of environmental regulation (ER), foreign direct investment (FDI), manufacturing industry agglomeration (MIA), knowledge intensive service industry agglomeration (KISA), and financial development (FD). The variables were measured as follows.

Environmental regulation (ER): it is usually divided into the formal and informal environmental regulation. This paper mainly considered the impact of formal environment on the efficiency of green innovation. Previous studies of cites at the prefecture level used SO_2_ removal rate as an indicator of environmental regulation at the city level. However, due to the change of the statistical caliber during the study period, we used the industrial smoke (dust) removal rate as an alternative indicator.

Foreign direct investment (FDI): to better smooth the volatility of the data, we used the city's FDI share of GDP for the year to represent it.

Manufacturing industry agglomeration (MIA): we used the manufacturing employment as the attribute value and measured the spatial Gini coefficient to express the manufacturing agglomeration. By calculating the location quotient of manufacturing industries in each city, we obtained the agglomeration level of the manufacturing industry.

Knowledge-intensive services industry agglomeration (KISA): according to the previous studies [51, 52], we selected the information, computer and software service, financial, leasing and business service, and education industries as the knowledge intensive industries. The agglomeration size is expressed by calculating the location quotient of the knowledge-intensive services in each city.

Financial Development (FD): It is expressed by the ratio of the sum of the loan balance and deposit balance of financial institutions in GDP at the end of the year.

### 3.3. Data Sources

This paper selected 286 prefecture level cities in China from 2005 to 2017 as the research object. The adjustment of administrative regions in the study period is based on the initial year. The data of GDP per capita, personnel engaged in scientific and technological activities, expenditure on science and technology and education, number of books per 100 people, number of Internet users, industrial waste gas emissions, industrial waste water emissions, industrial fixed waste emissions, and other data in the research came from the *China Urban Statistical Yearbook* and the *China Regional Economic Statistical Yearbook*. Partial missing data are supplemented by interpolation. The patent data are from the China Patent Bulletin network of the State Intellectual Property Office (http://epub.sipo.gov.cn/). The identification of the green patent is to obtain the number of green patents authorized at the prefecture level by matching, extracting, and screening patents one by one based on the IPC Green Inventory provided by the World Property Organization (WIPO) (https://www.wipo.int/classifications/ipc/en/) and the international IPC code of green patents.

## 4. Results

### 4.1. Time Evolution Trend

The feature of the efficiency structure of green innovation is: scale efficiency > pure technical efficiency > comprehensive technical efficiency. Factor input is the main source of efficiency, and technological progress is gradually becoming the driving force of efficiency improvement.  Figure 1 illustrates the decomposition characteristics of GIE. From 2005 to 2017, the overall efficiency evolution was scale efficiency > pure technical efficiency > comprehensive technical efficiency. The value of scale efficiency was between 0.46 and 0.66, which was always the maximum and the main source of comprehensive technical efficiency, while the pure technical efficiency value was between 0.36 and 0.48, which was at a low level. This showed that the current development of green innovation in China was still dominated by the increase of innovation elements, while the role of organization operation and system management in the process of green innovation was ignored. However, in recent years, the evolution trend of pure technical efficiency and comprehensive technical efficiency shows the same upward trend, while the scale efficiency shows a slight downward trend. A possible explanation is that China has implemented a stronger innovation-driven development strategy in recent years and has made a series of reforms to its science and technology innovation system.

The overall efficiency is low, rising in a high-low crisscross and showing the trend of Eastern rising, central collapse, and northeast stagnation. From the national point of view, the average value of green innovation efficiency was 0.283 and the highest value was 0.32, indicating that the overall GIE of cities is still at a low level. In terms of the time evolution, it experienced a process of rising in a high-low crisscross. The rapid growth from 2013 to 2017 was more significant, which indicates that the green economic transformation and the construction of ecological civilization have achieved preliminary results in China. From the regional point of view, the overall efficiency value of the eastern region was higher than that of the central and western regions, showing zonal spatial differentiation. Among them, the value of the central and western regions was lower than the national average, and the central region was slightly lower than that of the western region. This shows that most of the central and western regions are still dominated by “high energy consumption, high pollution, and low efficiency” industries. Besides, the evolution trend of the eastern, central, and western regions was basically the same and tended to rise in a high-low crisscross, especially in the eastern and central regions. On the contrary, the efficiency value of Northeast China has declined in recent years, from 0.219 in 2014 to 0.209 in 2017, which also echoes the stagnation of the economic growth in Northeast China in recent years.

### 4.2. Spatial Heterogeneity and Spatial Relevance of Urban GIE

The spatial heterogeneity of urban GIE was significant, and it was roughly staggered in height along the Hu Huanyong line.  Figure 2 shows the spatial distribution of green innovation efficiency in 2005 and 2017. On the whole, the spatial distribution of GIE was obviously uneven, with the Hu Huanyong line as the boundary, showing the characteristics of decreasing from southeast to northwest. The higher efficiency and relatively high efficiency mainly occurred in the eastern regions; the low efficiency and relatively low efficiency mainly occurred in cities in Guangxi, Yunnan, Guizhou, Gansu, Shaanxi, Jiangxi, Hunan, Hubei, and other provinces in the northwest China. The high-low unbalanced distribution pattern remained basically unchanged in two time periods, showing a strong local spatial dependence.

Urban GIE has significant spatial agglomeration and increasing innovation spillover effects. The Global Moran's I index was significantly positive at 1% level for the period from 2005 to 2017, which indicates that there was a positive spatial autocorrelation in GIE of cities and cities with higher or lower efficiency spatially were neighboring clusters. Temporally, the values of the Global Moran's I index were small during the period from 2005 to 2010, which indicates a weak spatial agglomeration during this time period; the increase was larger between 2011 and 2017, from 0.099 in 2011 to 0.28 in 2017, which indicates an increase in the spatial agglomeration of GIE among cities (Table 2).

The hot spots were evolving in clusters, and the mosaic characteristics of innovation agglomeration were increasingly strengthened.  Figure 3 shows the spatial distribution of hot and cold spots in 2005 and 2017. We can clearly find that the hot spots were distributed in Beijing, Tianjin, Hebei, Shandong, and areas in the Yangtze River Delta and Pearl River Delta. The central and western regions were generally cold spots, and there were no obvious high-value clusters. This was different from the spatial differentiation of green innovation efficiency, which shows that the spatial spillover effect of cities with high GIE in the central and western regions was limited. Furthermore, we find that the spatial dispersion of hot and cold spots did not vary much, which shows that the promotion of GIE was a relatively long-term process of technology accumulation. Besides, the regional innovation development and the industrial upgrading showed significant path dependence.

### 4.3. Decomposition of Urban GIE

In order to explore the sources of inefficiency in the internal input-output system, we decomposed the variables in the input-output system based on formula (3) and calculated the source and contribution rate of each variable's inefficiency decomposition with the help of Matlab2012a software platform (Table 3).

Input perspective: insufficient input in science and technology innovation personnel and public book collections per 100 people was the main source of inefficiency in most cities. From the decomposition of input inefficiency, the sources of inefficiency decomposition of cultural environment and innovation personnel were 0.423 and 0.435, respectively, and their contribution rates to the inefficiency were 22.65% and 23.31%, respectively, accounting for a high proportion in all input elements, which indicates that the innovation personnel and cultural environment were the main direction for improving the efficiency of the internal input-output system. From the perspective of vertical comparison, the contribution rate of science and technology innovation personnel inefficiency in the western and northeast regions was higher, which indicates that the urban green innovation development in these regions was facing a plight of insufficient innovative talents; however, the eastern regions had the largest contribution rate in the number of Internet users, which shows that compared with other regions, the eastern regions had an advantage in innovative talents but the innovation infrastructure still needs to be strengthened. The contribution rate of science and technology innovation personnel and number of Internet users in central China was more than 20%, which indicates that there was a large space for improvement in the investment of the innovative talents and innovation infrastructure in Central China.

Output perspective: excessive undesirable output and insufficient technological output were the main obstacles to improving the efficiency of urban green innovation. Among the sources of urban GIE inefficiency, the value of undesirable output reached 0.493 and the contribution rate in the whole output system reached 52.896%, followed by the inefficiency of technological outputs. The contribution rate of the undesirable output of the number of green patents granted at the national level was 44.311%. This shows that the current urban GIE is facing the dual constraints of excessive environmental pollution and weak technological progress. From a regional perspective, the environmental inefficiency of cities in the central and northeast regions was particularly serious, with a contribution rate of 57.145% and 54.915%, respectively, which was in line with the actual situation of the serious environmental pollution in the central and northeast regions; while in the western cities, the inefficiency caused by environmental pollution was relatively weak, but the lack of technological output was the primary factor leading to the inefficiency and the ineffective contribution rate reached 50.676%.

### 4.4. Spatial Econometric Regression Results

In this paper, Matlab2012a is used to estimate the regression results of spatial econometrics. The code of model operation comes from the code of spatial econometric model developed by Elhorst [49].The results of model estimation are shown in Tables 4 and 5. The selection of optimal interpretation model refers to the spatial panel econometric model test and selection framework proposed by Elhorst [49]. Firstly, the panel OLS regression without spatial effect is estimated, and the residual is tested. The results of LM Test has no spatial lag and robust LM Test also has no spatial lag test. For *P*=0, indicating that SLM and SEM models are more optimized than OLS regression. Then, the Wald spatial lag and Wald spatial error tests and LR spatial lag and LR spatial error tests were used. The results showed that the p value passed the 1% significance level test, indicating that SDM was the best explanation model. Furthermore, *P*=0 of Hausmann test significantly rejected the original hypothesis, indicating that fixed effects should be used. The results of LR-test spatial fixed effect and LR-test time-period fixed effect showed that the spatial and temporal double fixed effects should be used. Therefore, the final explanation of the model is the time and spatial double fixed effect of the spatial Durbin model.

The positive effect of FDI on the efficiency of urban GIE indicates that the sufficient capital, advanced technology, and management experience brought by FDI will have a certain demonstration effect on the local innovation subjects, so as to improve the efficiency of green innovation. The spatial lag coefficient was -0.1011, but it failed to pass the significance level test, which indicates that the spatial spillover effect of the foreign direct investment in local cities on proximity regions was negative, but not significant.

ER had no obvious effect on the efficiency of local green innovation, which shows that the policy tools and policy system of environmental regulation in China are not perfect and the backward effect on green innovation and the marginal effect of environmental improvement need to be improved. However, the spatial lag coefficient was 0.9841, reaching the significance level of 5%. This suggests that local ER has a positive spillover effect on GIE in neighboring cities, which is consistent with the findings of Pan et al. [53].

The empirical results show that the FD has a positive effect on urban GIE. FD is conducive to reducing the financing cost of innovation subjects, solving the problem of information asymmetry, optimizing the allocation of innovation resources and industrial structure, and improving the efficiency of green innovation. The regression coefficient of spatial lag was −0.1312, which was not significant. This shows that the spatial spillover effect of local FD on proximity cities is not significant.

The regression results show that the effect of KISA on urban GIE in both local and neighboring cities is not significant. The regression coefficient of KIS was 0.0349, and the regression coefficient of spatial lag was −0.1089, all failing to pass the significance level test. The possible reason was that in most cities, the correlation between the development of knowledge-intensive services industry and the green innovation technology was not high.

MIA has a positive effect on the urban GIE, showing that manufacturing industrial agglomeration is convenient for the information dissemination, division of labor and cooperation, sharing infrastructure and labor market, and the resulting technology spillover and operating cost reduction are conducive to the improvement of technological innovation efficiency. The spatial lag regression coefficient was 0.0776, not reaching the significance level, which indicates that the spatial spillover effect of local MIA on adjacent cities is not significant.

## 5. Discussion and Conclusion

In this paper, the GIE of Chinese cities was comprehensively evaluated by using the Undesirable-SBM model to construct the input-output index system of green innovation at the city level. The spatial-temporal evolution rules and influencing factors were revealed by using the exploratory spatial analysis and spatial econometric model. To sum up, the following main findings can be drawn:

1. Generally speaking, the GIE in Chinese cities is low and there is a large space for improvement. The feature of the decomposition of efficiency is scale efficiency > pure technical efficiency > comprehensive technical efficiency. The allocation of input-output of green innovation elements has not reached the optimal stage. However, from the perspective of evolution, the urban GIE in Northeast China is declining.
2. From the perspective of spatial evolution, the spatial differentiation of urban GIE evolves from polarization to equilibrium, with prominent Matthew effect. Cities with high or low efficiency are scattered on both sides of the Hu Huanyong line, and the changes of the urban quantity structure and spatial transition are small. In terms of spatial agglomeration, the Global Moran's I index fluctuates and the GIE tends to strengthen the agglomeration; however, the local hot and cold spots do not change much and the clustering of hot and cold spots shows the characteristics of spatial locking.
3. In terms of the structure of input-output system, the lack of investment in science and technology innovation personnel and innovation environment in the input system is the main source of inefficient investment in most cities. In the output system, the high output of environmental pollution and the lack of technological output are the main factors that restrict the promotion of urban GIE, especially in Central and Northeast China.
4. In terms of driving factors, the foreign direct investment, financial development, and manufacturing industry agglomeration have positive effects on the efficiency of urban GIE. However, the environmental regulation and the knowledge-intensive service industry agglomeration cannot promote the efficiency of GIE in most cities.

In the face of the serious ecological pollution, the Chinese government has made a huge commitment to promote green development. However, the results of this paper show that the level of green innovation efficiency in Chinese cities is still at a low level. Clearly, the findings of this paper have implications for policy formulation.

1. Considering the current situation that the overall GIE in Chinese cities is low, the proportion of pure technical efficiency is not high and the structure of green innovation input and output is still unreasonable, the Chinese government should adhere to the national strategy of the innovation-driven development and ecological civilization construction. In addition to the traditional innovation investment, the Chinese government should pay more attention to the reform of green innovation system. On the one hand, it is to complete the service system of green innovation and create an open, inclusive, collaborative, and efficient innovation environment. On the other hand, it is to cultivate more outstanding talents and improve the training mode and the evaluation and incentive mechanism for innovative talents.
2. The Chinese government should implement spatially differentiated environmental regulation policies and industrial policies, given that the current urban green innovation development patterns are inconsistent across different regions of China and that different socioeconomic factors operate differently on urban GIE. The current priority is to address the environmental pollution in Central and Northeast China and to increase the R&D investment and financial support to these cities, while the governments in the eastern and western regions should adopt stricter environmental regulation policies and improve the innovation infrastructure. At the same time, none of the governments should adopt a “one-size-fits-all” approach and a “herd effect” mode of following in the industrial upgrading and transformation; they should all focus on the development of industries that are compatible with the local innovation environment and the innovation capability of the cities. Only in this way can we achieve the coordinated and sustainable development of urban economy and environment.
3. Urban GIE has the characteristics of spatial agglomeration, but it also has obvious problems of the uneven regional development and the “Matthew effect.” This warns the Chinese government to pay attention to the uneven regional development of urban GIE. The government should strengthen its intervention in the technology trading market to avoid excessive concentration of innovation resources in a few cities; based on such an idea, the government should promote interregional innovation cooperation among innovation agents such as universities, research institutions, and enterprises and establish cross-regional platforms for innovation resource sharing and technology transfer; in addition to this, it should establish a counterpart innovation assistance system between regions, to promote the superior innovative cities to fund the less developed ones and encourage the docking cooperation between the eastern and the central-western and northeastern regions.

Although this paper provides new ideas for the study of urban GIE and explored its driving factors, there are still some limitations. On the one hand, for the measurement of urban pollutant emissions, we selected only the industrial pollution emissions. On the other hand, we captured only a portion of the urban GIE influencing factors. However, the measurement of green innovation efficiency is not only a question of whether the index selection is scientific and comprehensive but also about whether the evaluation method is accurate and reasonable. Therefore, further research is required to build a more comprehensive evaluation framework of green innovation efficiency, to explore the impact of more factors on green innovation efficiency and explain the spatial mechanism of the effect of these factors on green innovation efficiency in local and adjacent areas.

## Figures and Tables

**Figure 1:** Urban green innovation efficiency temporal evolution.

**Figure 2:** The spatial distribution evolution of urban GIE.

**Figure 3:** The evolution of hot spots and cold spots in urban GIE.

**Table 1:** Input-output indicator system of urban GIE.

Input- output structure	Variable layer	Index layer
Input variable	Capital input	Science and technology and education expenditure (input1)
	Labor input	Science and technology innovation personnel (input2)
	Innovation environment input	Public book collections per 100 people (input3)
Output variable		Number of internet users (input4)
	Technological output	Number of green patents granted (output1)
	Economic output	Per capita GDP (output2)
Undesirable output variable	Environmental pollution	Comprehensive environmental pollution index of industrial waste gas, industrial wastewater, and industrial fixed waste (bad-output)

**Table 2:** Global Moran's I index from 2005 to 2017.

	2005	2006	2007	2008	2009	2010	2011	2012	2013	2014	2015	2016	2017
Global Moran's *I*	0.083	0.091	0.053	0.067	0.106	0.146	0.099	0.0854	0.116	0.147	0.206	0.211	0.28
*Z*	3.882	6.768	3.938	4.859	7.84	10.807	7.468	6.294	8.487	10.879	15.011	15.419	20.501
*P*	0	0	0	0	0	0	0	0	0	0	0	0	0

**Table 3:** The inefficient decomposition sources and its contribution rate.

	Region	Science and technology and education expenditure	Science and technology innovation personnel	Public book collections per 100 people	Number of Internet users	Number of green patents granted	Per capita GDP	Environmental pollution
Inefficient value	The whole country	0.356	0.423	0.374	0.435	0.413	0.026	0.493
	Eastern China	0.321	0.338	0.373	0.453	0.306	0.017	0.366
	Central China	0.409	0.440	0.344	0.454	0.421	0.033	0.606
	Western China	0.284	0.421	0.343	0.375	0.510	0.031	0.466
	Northeast China	0.409	0.493	0.438	0.460	0.414	0.024	0.533

Contribution ratio	The whole country	19.047%	22.648%	20.037%	23.310%	44.311%	2.793%	52.896%
	Eastern China	17.915%	18.824%	20.789%	25.265%	44.398%	2.434%	53.168%
	Central China	20.934%	22.550%	17.616%	23.264%	39.740%	3.115%	57.145%
	Western China	17.243%	25.561%	20.811%	22.750%	50.676%	3.032%	46.291%
	Northeast China	19.679%	23.733%	21.049%	22.109%	42.637%	2.448%	54.915%

**Table 4:** Nonspatial effects model regression results and related test results.

	OLS	Spatial fixed	Time fixed	Spatial and time fixed
FDI	0.071^*∗∗∗*^	0.013	0.072^*∗∗∗*^	0.015
	(9.994)	(1.383)	(10.391)	(1.61)
ER	−0.104^*∗∗∗*^	−0.013	−0.092^*∗∗*^	−0.014
	(−2.6)	(−0.403)	(−2.47)	(−0.441)
FD	0.619^*∗∗∗*^	0.106^*∗*^	0.637^*∗∗∗*^	0.168^*∗*^
	(18.292)	(1.669)	(19.189)	(2.372)
KISA	−0.008	−0.096^*∗∗∗*^	−0.077^*∗∗*^	0.032
	(−0.25)	(−3.233)	(−2.224)	(0.921)
MIA	0.178^*∗∗∗*^	0.167^*∗∗∗*^	0.085^*∗∗∗*^	0.148^*∗∗∗*^
	(8.018)	(3.919)	(3.606)	(3.509)
Intercept	−0.621^*∗∗∗*^			
	(7.395)			
R2	0.206	0.010	0.235	0.006
sigma^2	0.037	0.043	0.090	0.040
LM spatial lag test	369.587^*∗∗∗*^	1375.605^*∗∗∗*^	74.276^*∗∗∗*^	61.860^*∗∗∗*^
LM spatial error test	955.253^*∗∗∗*^	1318.354^*∗∗∗*^	110.418^*∗∗∗*^	60.867^*∗∗∗*^
Robust LM spatial lag test	67.156^*∗∗∗*^	60.572^*∗∗∗*^	2.491	1.444
Robust LM spatial error test	652.822^*∗∗∗*^	3.321^*∗∗∗*^	38.633^*∗∗∗*^	0.452
Wald spatial lag test	20.009^*∗∗∗*^			
Wald spatial error test	19.551^*∗∗∗*^			
LR spatial lag test	24.004^*∗∗∗*^			
LR spatial error test	23.692^*∗∗*^			

Note: *t* statistics in parentheses. ^*∗*^*P* < 0.05, ^*∗∗*^*P* < 0.01, and ^*∗∗∗*^*P* < 0.001.

**Table 5:** Regression results of the spatial Durbin model.

Variable	Coefficient	*t*-stat	*z*-probability
FDI	0.0256^*∗∗*^	2.5436	0.0110
ER	−0.0245	−0.7399	0.4594
FD	0.1526^*∗∗*^	1.9676	0.0491
KISA	0.0349	0.9646	0.3347
MIA	0.1083^*∗∗*^	2.3697	0.0178
W*∗*FDI	−0.1011	−1.0990	0.2718
W*∗*ER	0.9841^*∗∗*^	2.0431	0.0410
W*∗*FD	−0.1312	−0.4540	0.6499
W*∗*KISA	−0.1089	−1.6126	0.1068
W*∗*MIA	0.0776	0.3066	0.7591
W*∗*dep.var	0.7910	19.8280	0.0000
*R*	0.6764		
sigma^2	0.0423		

Note: ^*∗*^*P* < 0.05, ^*∗∗*^*P* < 0.01, and ^*∗∗∗*^*P* < 0.001.

## Data Availability

The raw data supporting the conclusions of this article will be made available by the authors.
